# CCDC88A Post-Transcriptionally Regulates VEGF *via* miR-101 and Subsequently Regulates Hepatocellular Carcinoma

This article has been retracted.

**DOI:** 10.3389/fimmu.2022.859331

**Published:** 2022-04-13

**Authors:** Qiongying Hu, Yuchen Li, Hongqing Chen, Hongyan Liao, Yong He, Qin Zheng

**Affiliations:** ^1^ Department of Laboratory Medicine, Hospital of Chengdu University of Traditional Chinese Medicine, Chengdu, China; ^2^ Department of Laboratory Medicine, West China Hospital of Sichuan University, Chengdu, China

**Keywords:** hepatocellular carcinoma (HCC), Girders of actin filaments (CCDC88A), vascular endothelial growth factor (VEGF), microRNA-101, malignant behavior, cancer stem-like cells (CSCs)

## Abstract

**Background:**

miR-101 is one of the most abundantly expressed microRNA (miRNA) and exerst a critical role in hepatocellular carcinoma (HCC) by targeting to 3’ -untranslated region (UTR) of Girders of actin filaments (CCDC88A) and Vascular endothelial growth factor (VEGF) mRNA, but the underlying molecular mechanism remains to be elucidated. This study aimed to investigate the potential role of CCDC88A on malignancies and stemness by regulating VEGF *via* miR-101 in HCC.

**Methods:**

Gene Expression Profiling Interactive Analysis (GEPIA) was employed to analyze the relevance of CCDC88A expression with prognosis in HCC. Tissue slides were performed to confirm the protein level of CCDC88A in HCC. Correlation between CCDC88A and VEGF was transcriptionally and post-transcriptionally detected, followed by evaluation of malignancies.

**Results:**

By employing Immunohistochemistry, we found CCDC88A protein was upregulated in HCC tissues, which is closely correlated to poor prognosis and survival rate. Employment of GEPIA revealed the positive correlation between CCDC88A and VEGF in HCC, but not in liver tissue. Silencing of CCDC88A in Huh-7 and SK-HEP-1 cells significantly decreased proliferation, cell cycle phases, migration, invasion, colony formation, and tumor formation. Introduction of miR-101 mimics specifically targeting CCDC88A and VEGF decreased protein levels of both CCDC88A and VEGFA. Notably, inhibition of miR-101 reversed the correlation between CCDC88A and VEGFA protein levels, indicating that CCDC88A and VEGF may exert as a miR-101 sponge. The addition of SKLB1002, a VEGFR2 inhibitor inhibited malignant behaviors, which was further inhibited by the introduction of miR-101 mimics, indicating that CCDC88A regulates malignant behaviors partially *via* regulating VEGF. Moreover, CCDC88A also promotes the stemness of cancer stem-like cells derived from HCC cells depending on VEGF modification.

**Conclusion:**

Taken together, our findings suggested that the miR-101/CCDC88A/VEGF axis could be a potential therapeutic target of HCC treatment.

## Introduction

Liver cancer is one of the leading causes of cancer-associated death all over the world, which presents a high morbidity and mortality rate (1, 2). Based on the identification of histological pathology, HCC accounts for 70-85% of cases of liver cancer (3). Although numerous improvements have been made in the diagnosis and treatment of HCC in the past several decades, the high death rate and poor prognosis are still large concerns due to the high recurrence and metastatic rate (4). Investigating the mechanisms underlying malignancies, including recurrence and metastasis may promote the improvement of limiting tumor malignant progression, improve the prognosis and survival of HCC patients. Although promising therapeutic targets for HCC have been found, including α7-nAChR (5) and α5-Nicotinic acetylcholine receptor (6), the five-year survival rate remains low, and novel therapeutic targets need to be developed.

CCDC88A is identified as a critical regulator of physiological and pathological processes. Despite its physiological roles, such as regulating the migration of various cells by modifying actin-binding protein Akt (5), CCDC88A is also a bona fide metastasis-related protein that regulates several signaling pathways triggered by diverse classes of receptors (6, 7). CCDC88A is widely involved in diverse biological processes such as cancer migration, tumor angiogenesis, tumor-stroma interaction during cancer progression, cancer invasion, epithelial wound healing, organ fibrosis, and tumor metastasis (8–11). CCDC88A is reported to be overexpressed in a wide range of cancer types, including colorectal, breast, esophageal, gastric, glioblastoma multiforme, lung, and hepatocellular carcinoma (6). In the context of HCC, CCDC88A is reported to positively regulate malignant behaviors, including proliferation, colony formation, tumor metastatic invasion, radioresistance, and chemoresistance (12, 13). Yu and colleagues presented that, in Huh-7 and HepG2 cells, knockdown of CCDC88A resulted in inhibition of PI3K/AKT/HIF-1α signaling pathway and suppression of glycolysis (13). It is also reported that, in primary HCC tissues, the expression of CCDC88A was significantly higher than that in adjacent tissues (14). Knockdown of CCDC88A was also found to suppress malignant behaviors, without knowing the exact mechanism.

In past decades, accumulating evidence suggests that the dysregulation of miRNAs was widely found in all kinds of cancers and the abnormal expression of miRNAs is closely related to the progression of cancers (15). In liver cancer, several miRNAs have been reported to modulate malignancies, including let-7, miR-200 family, miR-122, miR-1246 (16). miR-101 is known as a key regulator and closely regulate the progression of many tumors, including HCC, *via* post-transcriptionally regulating VEGF (17). In HCC cells, miR-101 targets CCDC88A mRNA 3’-UTR and thus suppresses HCC cell proliferation, migration, and invasion (18). Introduction of miR-101 mimics exerts similar effects on HCC malignancies with small interfering RNA (siRNA) targeting to CCDC88A mRNA, demonstrated the role of miR-101 is depending on regulating CCDC88A, without knowing the exact mechanism.

Angiogenesis is a crucial process in HCC development since vascular formation is essential for solid tumors. VEGF is a critical promoter of angiogenesis in primary liver tumors (19). Anti-angiogenic therapies, by aiming at VEGF (such as sorafenib, a specific inhibitor of VEGF tyrosine kinase receptor), have been developed as a novel therapeutic strategy for HCC (20, 21). In cholangiocarcinoma, miR-101 was found to regulate angiogenesis by directly targeting 3’UTR of VEGF mRNA and subsequently repressed VEGF gene transcription (17). Moreover, VEGF was reported to exert critical roles in regulating the stemness of cancer stem-like cells (CSCs), which is a sub-population of HCC and resulted in recurrence (22). This indicated that miR-101 may simultaneously target both 3’UTR of CCDC88A and VEGF mRNA.

In this study, given that miR-101 is one of the most abundantly transcripted miRNA in liver and primary HCC, we sought to examine the regulation between CCDC88A, VEGF, and miR-101 in HCC and to validate their impact on HCC malignancies and tumor progression.

## Material and Methods

### Clinical Tissue Samples and Immunohistochemical Staining

Our study included 90 patients (74 men, 16women; mean age 52.3 years; range 27-84), who were recruited from May 2006 and August 2013, acquired by Shanghai Outdo cooperation (Shanghai, China). This experiment was approved by the Medical Ethics Committee of the Shanghai Outdo Biotech Company and performed according to the ethical guidelines (ethics No.: YB M-04-08). All patients who survived from 3 to 7.2 years were confirmed by telephone and mail. The study items included age, gender, tumor size, and tumor-node-metastasis stage. Tissues were fixed in 10% formaldehyde, embedded in paraffin, cut into 1.5 mm in diameter and 4 μm in thick, and mounted on a slide. Hepatocellular carcinoma (LIHC) tumor tissue and adjacent tissue sections were stained for immunohistochemistry analysis. Slides were baked at 60°C for 2 h, deparaffinization with xylene, and then rehydrated, after being washed three times in 1×phosphate buffered saline (PBS). Then, the rehydrated slide was incubated with 3% hydrogen peroxide for 10 min in methanol to inactivate endogenous peroxidase activity and then blocked using 2.5% bovine serum albumin (BSA) dissolved in PBS against nonspecific binding sites for 30 min at room temperature (RT). Then anti-CCDC88A antibody (diluted in 1:200; Cat. No.: ab179481; Abcam, Cambridge, England) was added for overnight incubation at 4°C. The incubated slide was then rinsed three times in ice-cold PBS and incubated with a horseradish-peroxidase-conjugated antibody (diluted in 1:5000; Cat. No.: ab7090; Abcam) for 1h at RT. The slides were developed then with 3, 3’-diaminobenzidine solution for 2-5 min, washed briefly in running water, and imaged under a microscope (Olympus BX51; Olympus, Japan).

### Cell Culture, CSCs Enrichment and Treatment

All Human tumor and non-tumor cell lines were bought from American Type Culture Collection (ATCC Manassas, VA, USA). Human non-tumor liver cell line HepRG, hepatocellular carcinoma cell lines Huh-7 and SK-HEP-1, colorectal adenocarcinoma cell lines HCT116 and Caco-2, lung adenocarcinoma cell lines A549 and H1299 were all maintained in Dulbecco’s modified Eagle’s medium (DMEM, Life Technologies, Grand Island, NY, US), supplemented with 10% heat-inactivated fetal bovine serum (FBS, Gibco, Thermo Scientific Inc., Waltham, MA, USA) and incubated at 37°C /5% CO_2_. Every 3 days, the medium was refreshed and when the cells covered 80% of the dish bottom, they were suspended with 0.25% trypsin (Gibco, Thermo Scientific Inc., Waltham, MA, USA).

To obtain CSCs, Huh-7 and SK-HEP-1 cells were kept in DMEM/F12 (1:1) basal medium (HyClone) with the addition of 10 ng/ml human epidermal growth factor (EGF, Miltenyi Biotec GmbH), 20 ng/ml basic fibroblast growth factor (bFGF, Miltenyi Biotec GmbH), and 2% B27 (Millipore Corporation, USA), without serum for 14 days and the medium was half-refreshed every three days.

To stimulate CSCs, recombinant VEGF (100 ng/ml) was added for 72-hour incubation. An inhibitor of VEGFR2 (10 μmol/L) was added to inhibit protein function.

### GEPIA Database Analysis

GEPIA is a comprehensive web-based analysis tool that includes tumor and normal sample RNA sequencing data from The Cancer Genome Atlas (TCGA) and Genotype-Tissue Expression projects and provides analysis of the interactive relationship, functions, and prognostic value of gene expression in cancer and normal tissues. The mRNA expression level and prognostic predictive significance of the CCDC88A gene in LIHC, colon adenocarcinoma (COAD), and lung adenocarcinoma (LUAD) were determined in GEPIA. Moreover, gene expression correlation analysis was also conducted between CCDC88A and VEGFA by using the GEPIA database.

### RT-Quantitative PCR (RT-qPCR)

Total RNA was extracted from cells using TRIzol reagent (Life Technologies, Grand Island, NY, USA), and 1 μg of total RNA was used for reverse transcription (Roche, Basel, Switzerland). Complementary DNA (cDNA) was used as the template for 40-cycle amplification in ABI7500 (Applied Biosystems, Foster City, CA, USA). The expression of genes was normalized using β-actin mRNA as an internal standard by the comparative Ct method.

The primer pairs used were as follows; CCDC88A forward 5’- AGGAAATGGGACCAACCTTGA-3’ and reverse 5’- GTGCATTCTAAGTGAGGCATCAT-3’; VEGFA forward 5’- AGGGCAGAATCATCACGAAGT-3’ and reverse 5’- AGGGTCTCGATTGGATGGCA-3’; β-actin forward 5’- CATGTACGTTGCTATCCAGGC-3’ and reverse 5’- CTCCTTAATGTCACGCACGAT-3’.

### Western Blot Analysis

Cells were suspended and collected followed by two washes with 1ml chilled PBS and resuspended using total protein lysis buffer (RIBOBIO, Guangzhou, China) followed by being lysed using SoniConvert^®^ sonicator (DocSense, Chengdu, China) following the instructions of the manufacturer. A measure of 20 μg of total protein sample was mixed with 10 μl 5×SDS loading buffer and incubated for 10 min at 100°C for denaturation and fractionated on 6-12% gradient SDS-PAGE gel and transferred to PVDF membrane. Western blot was carried out with anti-beta actin antibody at 1:5000 dilution (mAbcam 8226, Abcam, Cambridge, England), anti-CHK2 (phosphor S33+S35) antibody (cat. No.: ab68267, Abcam, Cambridge, England) at dilution of 1:1000, anti-p21 antibody (cat. No.: ab109520, Abcam, Cambridge, England), anti-GIV antibody (cat. No.: ab179481, Abcam, Cambridge, England), anti-VEGFA antibody (cat. No.: ab1316, Abcam, Cambridge, England). An HRP-conjugated anti-rabbit IgG antibody was used as the secondary antibody (Abcam, Cambridge, England). Signals were detected using enhanced chemiluminescence reagents (Thermo Scientific, Waltham, MA, USA). In this experiment, we made β-actin as the internal reference.

### Flow Cytometry and Cell Sorting

Cells were washed, and stained using a monoclonal anti-CD133 antibody (rabbit, ab216323, 1:2000; Abcam, Cambridge, Massachusetts), and analyzed by flow cytometry using 3 laser Navios flow cytometers (Beckman Coulter, Brea, CA, USA).

### PI Staining

Cells were suspended and collected by centrifugation at 400 g for 5 min at 4°C. After three washes using ice-cold PBS, the cell pellet was suspended and fixed in 70% ice-cold alcohol overnight at 4°C. Then cells were washed with ice-cold PBS three times and suspended with 400 μL PI solution at a final concentration of 5μg/mL for 10 min in the dark. Then, cells were analyzed by flow cytometry using three laser Navios flow cytometers (Beckman Coulter, Brea, CA, USA).

### Animal Experiment

Four week-old male BALB/c nude mice were purchased from Sichuan Dashuo Laboratory Animal Center (Sichuan, China). All procedures were approved by the Medical Ethics Committee of the Chengdu University of Traditional Chinese Medicine. Huh-7 cells transfected with shScrambled (shScrambled group) or shCCDC88A (shCCDC88A group) were collected and adjusted to final concentration of 1×10^7^ cells/ml. 2×10^6^ cells were injected subcutaneously into the left flank of the mice for each group (n=4). Tumor formation was monitored every five days. Tumor volume (TV) was measured and calculated using the following formula: TV (mm^3^) = *a* ^2^ × *b* × 0.52, where *a* and *b* were the shortest and longest diameters, respectively (23). Mice were sacrificed after 30 days and tumor specimens were fixed in 4% paraformaldehyde, embedded in paraffin, and cut into 5-μm thick slides. The slides were then stained with hematoxylin and eosin.

### Statistical Analysis

Statistical analysis was performed using SPSS version 19.0 (IBM, Corp). Data are presented as the mean ± standard deviation. A two-tailed unpaired Student’s t-test was used for statistical analysis. ANOVA was performed to compare multiple groups with one variable followed by Tukey’s *post hoc* test. P<0.05 was considered to indicate a statistically significant difference. The experiments were repeated at least three times.

## Results

### CCDC88A Is Positively Correlated With VEGFA and Acts as the Oncogenic Promoter for LIHC Individuals

To investigate whether CCDC88A is correlated with poor prognosis in LIHC, the data of the cancer genome ATLAS (TCGA) and the genotype-tissue expression (GTEx) (GEPIA, http://gepia.cancer-pku.cn/index.html) was employed and the results revealed that the expression of CCDC88A is upregulated in LIHC tumor tissue normalized to normal liver tissues (**Figure 1A**), which is not observed in COAD and LUAD. Overall survival rate showed that the higher CCDC88A in the LIHC patients suggested the lower survival rate (**Figure 1B**), which was also observed in analyzing disease-free survival rate, but not in COAD (**Figure 1C**) or LUAD (**Figure 1D**).

**Figure 1:** Expression of CCDC88A in human cancers determined by GEPIA database. **(A)** The expression profile of CCDC88A in three major human cancers, including Liver hepatocellular carcinoma (LIHC), colorectal adenocarcinoma (COAD), and lung adenocarcinoma (LUAD). Overall survival analysis and disease-free survival analysis of CCDC88A in LIHC **(B)**, COAD **(C)**, and LUAD **(D)** were determined by employing GEPIA database.

By considering that VEGF is transcriptionally promoted *via* STAT3/GIV signaling pathway in non-small-cell lung cancer (24), we then further analyzed the correlation between CCDC88A and VEGFA, one of the main isotypes of VEGF in LIHC, COAD, and LUAD. The results showed that in LIHC, but not COAD or LUAD (cor=0.16, *P*=4e-04; cor=-0.0033, *P*=0.96, respectively), CCDC88A and VEGFA were significantly correlated (cor=0.4, *P*=8.9e-16) (**Figure 2A**). We also analyzed the correlation between CCDC88A and VEGFB and VEGFC in LIHC and found that VEGFB, VEGFC were both positively correlated to CCDC88A in LIHC and liver tissues (**Figure 2B**). Notably, in normal tissues of the liver, lung, and colon, there is no obvious correlation between CCDC88A and VEGFA. All these data indicated that CCDC88A and VEGF, especially VEGFA, may synergically act as oncogenic promoters in LIHC specifically. By considering the positive correlation of CCDC88A and VEGFA in LIHC, but not in Liver tissues, we further focused on the regulation of CCDC88A on VEGFA, but not VEGFB or VEGFC.

**Figure 2:** CCDC88A was positively correlated with VEGFA in LIHC. To analyze the correlation between CCDC88A and VEGFA, the GEPIA database was employed and the scatter plots show Pearson’s correlation of CCDC88A expression with expression of VEGFA. **(A)** The correlation between CCDC88A and VEGFA in LIHC, COAD, and LUAD was analyzed. **(B)** The correlation between CCDC88A and VEGFB or VEGFC in LIHC was analyzed.

To further confirm the upregulation of CCDC88A in LIHC, four pairs of liver cancer tissues and adjacent tissues were detected by performing immunohistochemistry. The results presented that positively stained cells of CCDC88A in cancer tissues are obviously higher than that in paired adjacent tissues (**Figure 3**).

**Figure 3:** Immunohistochemical staining of CCDC88A in serious LIHC and non-tumor adjacent tissues. Four pairs of LIHC tissues were Immunohistochemically analyzed. Images were taken under amplification of 2, 10, and 40, respectively.

### CCDC88A Affected Malignant Behaviors in Liver Cancer Cell Lines and Promoted Tumor Formation in Nude Mice

To further confirm the correlation between CCDC88A and VEGFA in cancer cell lines, the mRNA and protein levels of CCDC88A and VEGFA were evaluated in LIHC cell lines (Huh-7 and SK-HEP-1), COAD cell lines (HCT-116 and Caco-2), and LUAD (A549 and H1299), compared to non-tumor liver cell line HepRG. As it is shown in **Figure 4A**, both CCDC88A and VEGFA mRNA levels in Huh-7 and SK-HEP-1 were significantly higher than those in HepRG cells. Protein levels of CCDC88A and VEGFA were also observed to be upregulated obviously in LIHC cell lines (**Figure 4B**). Thus, we chose Huh-7 and SK-HEP-1 to study the synergic effect of CCDC88A and VEGFA in LIHC.

**Figure 4:** CCDC88A is positively correlated with VEGFA and regulates cell proliferation. **(A)** RT-qPCR was performed to detect the mRNA level of CCDC88A in cancer cell lines, including Huh-7, SK-HEP-1, HCT-116, Caco-2, A549, and H1299, compared with HepRG. *P < 0.05, vs. HepRG group. **(B)** Western blot was performed to detect CCDC88A protein in all these cell lines. After transfecting shRNA target to CCDC88A mRNA (shCCDC88A), compared to scrambled shRNA (shScrambled), CCDC88A mRNA was detected in both Huh-7 and SK-HEP-1 cells **(C)**, and protein level was measured by performing western blot **(D)** *P < 0.05, vs. shScrambled group. **(E)** 48 h after shCCDC88A transfection, cell cycle phase distribution was measured by performing PI staining followed by flow cytometric analysis. *P < 0.05, vs. shScrambled group.

To modify the expression of CCDC88A, we transfected shRNA target to CCDC88A mRNA (shCCDC88A) into Huh-7 or SK-HEP-1 and as it is illustrated in **Figure 4C**, shCCDC88A significantly decreased CCDC88A mRNA level in both of these cell lines. According to western blot results, it was observed that knockdown of CCDC88A simultaneously decreased VEGFA protein, indicating that CCDC88A may positively regulate VEGFA protein (**Figure 4D**).

CCDC88A was reported to tightly regulate malignant behaviors in several kinds of cancers, including in LIHC (18, 25, 26). We then evaluated the effect of efficiently knockdown CCDC88A on malignant behaviors in Huh-7 and SK-HEP-1 cells. As it is shown in **Figure 4E**, and as expected, CCDC88A knockdown significantly arrested the cell cycle at G_1_/G_0_, indicating its cell proliferation promoting effect. We also detected cell viability (**Figure 5A**), migration (**Figure 5B**), invasion (**Figure 5C**), colony formation (**Figure 5D**), and tumor formation in soft agar (**Figure 5E**), consistently, it is presented that in both two cell lines, knockdown of CCDC88A remarkably decreased all these malignant behaviors.

**Figure 5:** Knockdown of CCDC88A inhibits malignant behaviors in Huh-7 and SK-HEP-1 cells. After 48-h transfection, malignant behaviors of Huh-7 and SK-HEP-1 cells were detected, including cell viability **(A)**, migration **(B)**, invasion **(C)**, colony formation **(D)**, and tumor formation in soft agar **(E)**. *P < 0.05, vs. shScrambled group.

To further evaluate its effect in promoting tumor growth, Huh-7 with or without CCDC88A silencing was grafted in nude mice. As it is shown in **Figures 6A–C**, CCDC88A silencing significantly inhibited tumor formation in nude mice compared to those transfected using shScrambled RNA, further demonstrating that CCDC88A exerts a critical role in promoting tumor growth *in vivo*.

**Figure 6:** CCDC88A knockdown decreased tumor formation in nude mice. **(A)** 30 days after injection, grafting tumors were obtained and the tumor size of each mouse was measured every five days. N=4 for each group. *P < 0.05, vs. shScrambled group; **P < 0.01, vs. shScrambled group. **(B)** Body weight of each mouse was measured every five days. **(C)** H&E staining in each grafting tumor was imaged.

### CCDC88A mRNA May Protect VEGFA mRNA From Post-Transcriptional Regulation by miR-101

miR-101 is considered to play a critical role in HCC (18), potentially *via* downregulating CCDC88A by binding to CCDC88A mRNA 3’-UTR. Notably, in HCC, it is also reported that miR-101 binds to VEGF mRNA 3’-UTR and thus inhibits angiogenesis (17), which indicated that the positive correlation between CCDC88A and VEGFA may be due to post-transcriptional regulation of miR-101. To confirm whether CCDC88A and VEGFA protein levels were regulated by miR-101 specifically, we employed miR-4448 and miR-150-5p, which were reported to target CCDC88A (27) or VEGFA (28) mRNA, respectively. We efficiently introduced miR-101, miR-4448, or miR-150-5p mimics respectively into Huh-7 and SK-HEP-1 cells (**Figure 7A**). The introduction of miR-101 significantly decreased both CCDC88A and VEGFA protein levels (**Figure 7B**). Notably, introduced miR-4448 or miR-150-5p mimics significantly decreased CCDC88A and VEGFA simultaneously, indicating that the correlation of CCDC88A with VEGFA is potentially dependent on the post-transcriptional regulatory mechanism, such as acting as miR-101 sponge for each other (**Figure 7B**). Introduced miR-101 antagonist abolished the decrease of VEGFA after miR-4448 mimics introduction, and the decrease of CCDC88A after miR-150-5p mimics introduction (**Figure 7C**), which demonstrated that the presence of miR-150-5p is critical for the correlation of CCDC88A with VEGFA.

**Figure 7:** CCDC88A may protect VEGFA from miR-101 posttranscriptionally. **(A)** After transfection of miR-101, miR-4448 or miR-150-5p mimics for 48 h, respectively, miR-101, miR-4448, or miR-150-5p RNA levels were detected by performing RT-qPCR. **(B)** After transfection of miR-101, miR-4448 or miR-150-5p mimics for 48 h, respectively, protein levels of CCDC88A and VEGFA were detected by performing western blot. *P < 0.05, vs. NC group. **(C)** miR-4448 or miR-150-5p was co-transfected into Huh-7 and SK-HEP-1 cells together with different concentrations of anti-miR-101 antagonist (25, 50, or 100 nM), and protein levels of CCDC88A and VEGFA were detected by performing western blot. *P < 0.05, vs. NC group.

### CCDC88A Mainly Contributes to Promoting Malignancies, but Not VEGFA in HCC

To identify whether CCDC88A contributes to promote malignancies in HCC *via* regulating VEGFA, we added SKLB1002, a VEGFR2 inhibitor, with or without CCDC88A knockdown in Huh-7 and SK-HEP-1 followed by detecting malignancies. As it is shown in **Figure 8A**, blockage of VEGFA obviously decreased cell proliferation, and simultaneous knockdown of CCDC88A further decreased cell proliferation, potentially *via* inducing cell phase blockade at G_1_/G_0_ (**Figure 8B**). Knockdown of CCDC88A resulted in an increase of p21 and p-CHK2 protein levels, which are two key regulators of cell cycle progression (**Figure 8C**).

**Figure 8:** CCDC88A regulates cell proliferation partially *via* regulating VEGFA. **(A, B)** After the addition of SKLB1002, a VEGFR2 inhibitor, transfected miR-101 mimics further blocked the cell cycle at G_1_/G_0_. *P < 0.05, vs. mock group; *P < 0.05, vs. SKLB1002/NC mimics group. **(C)** western blot was performed to detect p-CHK2 and p21 protein levels. *P < 0.05, vs. SKLB1002/NC mimics group.

We then also assessed the contribution of CCDC88A knockdown, while SKLB1002 was added, on migration, invasion, colony formation, and tumor formation in soft agar. As is shown in **Figures 9A, B**, the addition of SKLB1002 significantly decreased migration and invasion, and the knockdown of CCDC88A failed to further affect these behaviors. Interestingly, knockdown of CCDC88A successfully further decreased colony formation and tumor formation in soft agar, which was significantly inhibited by the addition of SKLB1002 (**Figure 9C**). Taken together, CCDC88A may mainly contribute to the regulation of malignant behaviors, which is partially *via* upregulating VEGFA.

**Figure 9:** CCDC88A regulates malignant behaviors in Huh-7 and SK-HEP-1 cells partially *via* regulating VEGFA. After the addition of SKLB1002, a VEGFR2 inhibitor, transfected miR-101 mimics further inhibited malignant behaviors including migration **(A)**, invasion **(B)**, and colony formation **(C)**.

### CCDC88A Regulates Stemness *via* Promoting VEGFA in HCC Derived Stem-Like Cells (CSCs)

By considering that VEGF accelerates the recurrence and promotes stemness in hepatocellular carcinoma (22), we evaluate whether CCDC88A promotes stemness of CSCs derived from Huh-7 and SK-HEP-1 cells. As shown in **Figure 10A**, CCDC88A knockdown decreased spheres formed by being cultured in serum-free medium, and the addition of recombinant VEGF increased spheres despite CCDC88A silencing, which indicates the inhibitory role of CCDC88A knockdown on sphere formation was remarkably reversed by VEGF stimulation. CCDC88A silencing significantly decreased cell viability, which is not reversed by the addition of VEGF (**Figure 10B**). To further confirm the inhibitory effects of CCDC88A on stemness, but not only on cell proliferation, we measured Nanog and CD133, which were reported to be positively regulated by VEGF in hepatocellular CSCs (22). Expectedly, knockdown of CCDC88A significantly decreased Nanog and CD133 expression, which was reversed by the addition of VEGF. Notably, the addition of VEGF significantly increased Nanog and CD133 expression, demonstrating that CCDC88A regulates stemness of CSCs mainly dependent on modifying VEGF (**Figure 10C**).

**Figure 10:** CCDC88A regulates stemness of CSCs *via* modifying VEGF. **(A)** After CCDC88A silencing with or without VEGF addition, sphere formation of Huh-7 and SK-HEP-1 in serum-free medium was collected. **(B)** After CCDC88A silencing with or without VEGF addition, cell viability was measured by performing CCK-8. *P<0.05, vs. shScrambled group. **(C)** After CCDC88A silencing with or without VEGF addition, expression of Nanog and CD133 were semi-quantitatively analyzed by western blot.

## Discussion

Our study showed that CCDC88A is upregulated in LIHC and positively correlated with the expression of VEGF. The vascular endothelial growth factor (VEGF) family which exerts a large role in the regulation of angiogenesis, is comprised of five isotypes (VEGFA, VEGFB, VEGFC, VEGFD, and PIGF). In this study, we analyzed the correlation of CCDC88A and VEGFA, VEGFB or VEGFC, in LIHC tissues, and interestingly found that VEGFA, but neither VEGFB nor VEGFC, is positively correlated with CCDC88A, which indicated the potential interaction between CCDC88A and VEGFA. Knockdown of CCDC88A by introducing shRNA target to CCDC88A mRNA expectedly inhibited malignant behaviors in both Huh-7 and SK-HEP-1 cells, including cell proliferation, migration, invasion, colony formation, and tumor formation. Interestingly, miR-101 was found to target CCDC88A mRNA 3’UTR and VEGF mRNA 3’UTR, respectively. We then presented that high CCDC88A mRNA level is positively correlated with VEGFA mRNA level, and CCDC88A promotes malignant behaviors, at least partially, *via* the presence of VEGFA/VEGFR2 signaling. Taken together, we hypothesize that CCDC88A and VEGF may protect each other from miR-101, and thus promotes malignant behaviors in HCC cells.

miR-101 is a downregulated miRNA in HCC tissues and its expression was negatively associated with a poor prognosis of HCC patients (29). By targeting several oncogenes, such as Enhancer of Zeste 2 Polycomb Repressive Complex 2 Subunit (EZH2), Dual-specificity phosphatase (DUSP), Myeloid cell leukemia-1 (Mcl-1), miR-101 exerts as a tumor suppressor. However, the regulatory roles of miR-101 on CCDC88A and VEGFA in HCC have not been fully illuminated. In this study, we focused on the regulatory role of miR-101 on CCDC88A and VEGFA. By introducing CCDC88A specific miR-4448 or VEGF specific miR-150-5p, it is illustrated that specific knockdown of CCDC88A or VEGF mRNA, also relatively decreased VEGF or CCDC88A level. The interference between CCDC88A and VEGF can be eliminated by inhibition of miR-101 *via* introducing antagonist miR-101, indicating that the positive correlation between CCDC88A and VEGF is potentially *via* the presence of miR-101. Inhibition of the VEGFR2 signaling pathway can inhibit the malignant behavior of HCC cells, while miR-101 mimics can further inhibit the malignant behavior of HCC cells, suggesting that CCDC88A partially regulates the malignant behavior of HCC cells through VEGF. All these results indicate that a relatively high level of miR-101 may exert an anti-tumor effect in HCC. Also, by considering that miR-101 is widely reported to be downregulated in HCC tissues (29), it indicated the critical role of the mechanism of activating endogenous miR-101. However, in this study, it was failed to be evaluated, which is one of this study’s limitations.

The VEGF family of proteins mainly comprises VEGFA, VEGFB, VEGFC, VEGFD, and PIGF (30). VEGFA is one of the best-featured family members of the VEGF family, which are most strongly stimulated by the angiogenesis process, and therefore be considered as a promising target in numerous anti-cancer treatments (31). VEGF-A is secreted by many cell types, such as endothelial cells, fibroblasts, smooth muscle cells (32), platelets (33), neutrophil (34), macrophages (35), and about 60% of all tumors (36). By employing the GEPIA database, the correlation between CCDC88A and VEGFA/VEGFB/VEGFC was analyzed and only CCDC88A and VEGFA were found to be positively correlated specifically in LIHC tissues, but not in normal liver tissues. miR-101 was reported to target 3’UTR of VEGF mRNA and subsequent repressed VEGF gene expression in cholangiocarcinoma (17). This indicates that miR-101 may exert a similar role in other kinds of cancer. It is also possible that miR-101 exerts different roles in different kinds of cancer by targeting different targets. Although it was presented in this study that miR-101 specifically targets VEGF, it is still largely unknown how VEGFB and VEGFC correlate with CCDC88A differently.

In conclusion, this study of CCDC88A in HCC has demonstrated the significant predicting effect of CCDC88A levels on malignancies and survival of HCC patients. Our results indicate that CCDC88A and VEGF are positively correlated in HCC cells *via* the presence of miR-101, and thus identified CCDC88A and VEGF as the promising prognostic biomarkers of HCC. Taken together, upregulation of CCDC88A and positively correlated VEGF may act as the biomarkers in the diagnosis and treatment of HCC.

## Data Availability Statement

Datasets presented in this study can be found in online repositories. The names of the repository/repositories and accession number(s) can be found in the article/**Supplementary Material.**

## Ethics Statement

The animal study was reviewed and approved by the Medical Ethics Committee of the Chengdu University of Traditional Chinese Medicine.

## Author Contributions

QH and QZ designed the experiments and performed molecular-related experiments in this study. QH, YL, and HC performed experiments on processing cells. QH, YL, HL, and YH are responsible for data collection and performed the statistical analysis. HL and QZ wrote the manuscript. QZ revised manuscript. All authors read and approved the final manuscript.

## Funding

The Technical Innovation Research and Development Project of Scientific and Technological Office of Chengdu (2021-YF05-01726-SN), the Science and Technology Project of the Health Planning Committee of Sichuan Project (No. 18ZD039).

## Conflict of Interest

The authors declare that the research was conducted in the absence of any commercial or financial relationships that could be construed as a potential conflict of interest.

## Publisher’s Note

All claims expressed in this article are solely those of the authors and do not necessarily represent those of their affiliated organizations, or those of the publisher, the editors and the reviewers. Any product that may be evaluated in this article, or claim that may be made by its manufacturer, is not guaranteed or endorsed by the publisher.
